The article "Guide to the design and application of online questionnaire surveys" was published in 2016. Journal: Nepal J Epidemiol.

#  Guide to the design and application of online questionnaire surveys 

**DOI:** 10.3126/nje.v6i4.17258

**Published:** 2016-12-31

**Authors:** Pramod R Regmi, Elizabeth Waithaka, Anjana Paudyal, Padam Simkhada, Edwin van Teijlingen

**Affiliations:** 1 Faculty of Health and Social Sciences, Bournemouth University, England UK.; 2 Visiting Research Fellow, Chitwan Medical College (CMC), Tribhuvan University Nepal.; 3 The School of Environment, Charles Darwin University, Darwin Australia.; 4 Faculty of Education, Health and Community, Liverpool John Moores University UK; 5 Manmohan Memorial Institute of Health Sciences, Tribhuvan University, Nepal.; 6 Nobel College, Pokhara University, Nepal.

**Keywords:** Online surveys, Internet survey, Web based survey, Questionnaire design, Research methods, Research ethics

## Abstract

Collecting research data through traditional approaches (face-to-face, postal or telephone survey) can be costly and time consuming. The emerging data collection approach based on internet/e-based technologies (e.g. online platforms and email), is a relatively cost effective survey alternative. These novel data collection strategies can collect large amounts of data from participants in a short time frame. Similarly, they also seem to be feasible and effective in collecting data on sensitive issues or with samples they are generally hard to reach, for example, men who have sex with men (MSM) or migrants. As a significant proportion of the population currently in the world are digitally connected, the shift from postal (paper-pencil) or telephone towards online survey use in research is in the interests of researchers in academia as well as in the commercial world. However, compared to designing and executing paper version of the questionnaire, there is limited literature to help a starting researcher with the design and a use of online questionnaires. This short paper highlights issues around: a) methodological aspect of online questionnaire survey; b) online survey planning and management; and c) ethical concerns that may arise while using this option. We believe that this paper will be useful for researchers who want to gain knowledge or apply this approach in their research.

## Introduction

Questionnaire surveys are a popular data collection method for academic or marketing research in a variety of fields. Face-to-face, telephone interviews and postal surveys are traditional approaches of completing questionnaire surveys. However, with the growing access to the internet facility globally [ 1,  2 ], for example, internet penetration in Nepal, a low-income country, increased exponentially in the past two decades, from less than 50 users in 1995 to 11.9 million users (about 45% of total population) in 2015 [ 3 ] and the price of technology devices (e.g. tablet computers, hardware) and software continuing to reduce [ 4 ], an novel internet-based data collection technique such as online questionnaire survey has become popular in recent years [ 5 ]. Recently, qualitative data collection through online focus groups is also emerging [ 6, 7 ], suggesting, research participants in the digital age can now interact with each other and the interviewer/facilitator in an online- multimedia setting. 

 Data collection through an online survey appears to have the potential to collect large amounts of data efficiently (i.e. with less error due to the lack transferring written data on to a computer), economically (as it requires low human resource efforts while collecting or managing data) and within relatively short time frames. Online survey approach is also very useful when collecting data from hard-to-reach populations such as lesbian, gay, bisexual and transgender (LGB&T) or travellers, etc. Moreover, people with certain conditions, such as HIV are often hard to access since they are stigmatized offline [ 4 ]. Studying these sub-populations can be possible through an online survey approach as this may help access these hard to reach population by sending an invitation through a range of media and discussion platforms (e.g. social media, discussion fora).

Online survey approach provides convenience in several ways, for example, a) respondent can answer at a convenient time; b) respondent can take as much time as they need to response questions; c) respondent can complete survey in multiple sessions. Similar to the paper-based survey; online questionnaire surveys are capable of question diversity (e.g. dichotomous questions, multiple-choice questions, scales), skip irrelevant questions for sub-groups in the sample (i.e. no pregnancy questions for men) and even collect an open-ended questions (qualitative data) through a free text box. Similarly, the construction of the online questionnaire can also be built to help better response rate for each item; for example, respondents must answer a question before advancing to the next question. This, however, might create an unfavourable situation to some research participants if they do not want to answer sensitive questions such as sexual behaviours or drug use. Unlike the paper postal survey, through this approach, follow up could be easy through email which enhance response rate. 

 There is substantial evidence that many large cross-country studies have been completed using online questionnaire surveys through popular dedicated platform (e.g. https://www.surveymonkey.co.uk/, https://www.onlinesurveys.ac.uk/about/ , https://www.qualtrics.com/ ).These platforms allow researchers to deploy and analyse surveys via the web without any advanced technical knowledge. Despite these developments, there is not much research focusing on an online survey or other technology-based survey methodologies, simply because they have been introduced a few years ago. 

 An online survey questionnaire survey follows the same characteristics as the paper version of the survey. However, the data collection strategies have specific characteristics (e.g. technological, demographic, response rate) that affect their design and implementation. Online questionnaires can only produce valid and meaningful results if the: a) layout of the questionnaire and all its questions/items are clear and precise; b) if they are appropriately executed (for example, completing survey through a mobile app or via tablet might attract young generation but may not work well with elderly population); and c) if they are asked consistently across all respondents. Therefore, a careful consideration needs to be given while designing the online questionnaire survey. In this paper, we discuss: a) methodological aspect of online questionnaire survey; b) online survey planning and management; and c) ethical concern that may arises while using this option.

## Methodological components

Whilst developing and operationalising the online questionnaire survey, six methodological components are critical to successful online surveys. These are (a) user-friendly design and layout; (b) selecting survey participants; (c) avoiding multiple responses; (d) data management; e) ethical issues; and f) piloting tools. These are discussed below.

### a) User-friendly design and layout

Generally, online survey link is promoted through an email, websites, social media or online discussion plateforms and potential survey participants are invited to take part the survey. Research participants always prefer a tool which is easy to follow and complete. The format of the questionnaire, therefore, should be easy for the participants to navigate around and should need only a minimum of computer skills for their completion. The items should be short, clear and easy to read by the participants, e.g. elderly people might need larger fonts. Similarly, research participants may be more open to sharing sensitive or personal information such as age, sex, after completing other questions, sensitive or personal questions should be placed at the end. Dillman [ 8 ] found that visual presentation is essential and also strengthen response rates, lead to longer download times of large files (especially in a setting where internet speed is slow) and this must be considered. Moreover, as online surveys are generally self-administered, answering instructions must be extremely clear.

### b) Selecting survey participants

An easy access to surveys for all participants is essential in any online questionnaire survey [ 9 ]. Therefore, an online questionnaire may be appropriate only for a certain age groups. [ 10 ]. For example, an online study among elderly population would not be appropriate if the proportion of elderly who access/use internet is low. Similarly, if the survey link is promoted through social media (e.g. Twitter, Facebook), it might not capture the views from other people who do not use social media. In such circumstances the survey should be promoted through other channels and perhaps other possible data collection strategies (e.g. telephone or paper survey) should be combined with your online survey. Although, relatively little may be identified about the background characteristics of people in online communities, except basic demographic variables, and tracking non-response rate is not an easy in most online survey [ 5,  11 ], it is very likely that participants in online surveys are more experienced or have stronger internet skills. They may be younger male and from households having fairly high incomes [ 12 ], however, with the modernisation and wide coverage of the internet facilities globally (particularly through mobile phones), recently the gap in internet use has decreased in countries like Nepal.

### c) Avoiding multiple responses

Another important feature of the online survey design is the ability to avoid multiple responses. This is a particularly challenging when incentives are provided to the survey participants. In order to minimise this problem, online survey design should able to include a feature that enables to register interested participants (through their email) in the first stage so that the online tool will be able to assign a unique participant number which will minimise the chance of multiple enrolments into the study. A personalised link to access the online questionnaire can be sent to participants’ email address. It is very important that the email should be used for sharing the survey link only (to ensure participant’s details are protected). Restriction through an IP address could be another strategy to avoid multiple enrolments; however, it limits the opportunity for participants (e.g. family members or students living in communal dwelling) who share a common IP address. Similarly, participants should be offered completing the survey across multiple sessions if they wish (as long as they use the same device), as survey responses save automatically as participants progress through the survey pages.

### d) Data management

Generally online survey platforms offer convenient and reliable data management. By design, online survey format protects against the loss of data and facilitates data transfer into a database (e.g. excel or SPSS) for analysis [ 9,  10 ]. As these approaches provide the ability to export responses into a compatible database, it eliminates transcription errors and prevents survey modification by the survey participant. It can be argued the overall ease of use for well-designed questionnaires for both study participants and the researchers potentially improves the reliability and validity of the data collection process and the collected data [ 13 ].

### e) Ethical issues

Online administration of surveys raises unique ethical questions regarding key ethical components including:

#### i. Informed consent

In most online survey tools, it is not possible to explain the study or to take verbal consent from participants. Researchers therefore have turned to ensuring that all information regarding the study, participants' rights and researcher's contact details are provided on the first page of the survey [ 14 ]. However, this is dependent on the study design. For example, in the conduct of e-Delphi studies, researchers have the option to administer participant information sheets, consent forms and additional study information by personal contact thereby allowing for oral consent [ 15 ]. The consent practice needs to be cautiously considered and determined. One increasingly common way is presenting items as would be found on paper-based consent forms such that the items must be endorsed before the next page can be opened.

#### ii. Privacy and confidentiality

There have been concerns regarding the ability of online administration tools ability to facilitate privacy and confidentiality [ 16 ]. Most of these tools rely on the researchers' ingenuity in setting up the survey settings to limit for instance participants' IP addresses. However, tools such as Survey Monkey have been associated with easily accessible data from surveys shared from a common account thereby compromising confidentiality [ 14 ].

#### iii. Right to withdrawal or omission of items

Study participants should have a right to withdrawal from the survey in addition to the choice to opt out of sharing the data already provided on an online questionnaire. Researchers should, therefore, ensure that the opportunity to erase or skip questions or backtrack through the survey is provided in order to maintain ethically sound research conduct. As a rule, only items relating to the consent form should require a response [ 14 ].

### f) Piloting

When the survey tools, contents, platforms are decided, it is very important to carry out a pilot [ 17,  18 ] with potential participants. Pilot studies can help ensure the adequacy of the questions, ordering of the questions, comprehensiveness of the contents, instructions are clear and adequate, feasibility of the technology (e.g. download time), skipping patters, data compatibility/transfer issues etc. Not all piloting has to be online as researchers can conduct cognitive interviews with those involved in a pilot study, although obviously certain aspects such as download time require piloting an electronic version of the survey.

## Conclusion

Internet access is increasing across the globe has resulted in an increase in the use of online surveys. This data collection approach has a potential to collect both qualitative and quantitative data. Conducting an online survey enables access to large and geographically distributed populations. Experts have argued it as a cost-effective and time saving for the researcher. Although multiple data collection strategies help achieve a better response, combining email, postal and web-based survey, may, however, prove impractical or financially unfeasible to use. If designed and executed rigorously, results from an online survey may be no different than paper based survey results, yet may demonstrate to be advantages due to lower costs and speedy distribution. When designing an online survey, researchers should consider a number of principles such as simplicity in items included, feasibility, appropriateness of online surveys for the target participants, being culturally and ethically sensitive, completeness and neutrality. Adhering to these principles will ensure that your online survey is methodological sound.
